The article "Bayesian Estimation of Supply Chain Innovation Path" was retracted in 2023. Reasons: unreliable results or conclusions; concerns about the data; concerns about the peer review; concerns about the citations.

# Bayesian Estimation of Supply Chain Innovation Path

**DOI:** 10.1155/2022/3738867

**Published:** 2022-06-16

**Authors:** Xin Zhang, Jian He, Weiguo Tian

**Affiliations:** ^1^Business College, Jiaxing University, Jiaxing 314001, Zhejiang, China; ^2^Pinghu Normal College, Jiaxing University, Jiaxing 314001, Zhejiang, China; ^3^Zhejiang Wanli University, Ningbo 315100, Zhejiang, China

## Abstract

With the transformation of the supply chain from factor driven to investment driven and to innovation driven, supply chain innovation has attracted more and more attention. This paper obtains the Bayesian prior probability of innovation and studies the supply chain innovation path from the perspective of strategy and behavior. The model divides the overall innovation capability of the supply chain into specific node tasks and assets (Capability Set), and the innovation demand of the supply chain is expressed in the form of the conditional probability of market demand. Under the conditions of minimum risk, minimum cost, and rapid market response, it determines who should lead the supply chain innovation first and what type of supply chain innovation should be carried out first. Finally, taking the supply chain of the professional market in Zhejiang Province as an example, this paper verifies the theoretical model of supply chain innovation decision-making. The innovation of the supply chain of Zhejiang's specialized market is decomposed into the capability set of each enterprise node of the supply chain. This paper transforms the group innovation ability of the supply chain in the professional market into the individual innovation ability of a single enterprise node and reveals the starting point and intensity of the demand innovation of products/services in the supply chain.

## 1. Introduction

The rise of the antiglobalization trend of thought has brought serious negative effects on the global industrial chain and supply chain. Global industrial chain supply chain would be quickly reshaped. In terms of the industrial chain, many countries were more sensitive to the safety of the industrial chain after the test of epidemic situation, and developed countries will accelerate the “industrial return.” In the supply chain, some enterprises will consider sacrificing a part of profits, reducing the investment scale in a single market, and laying out the supply chain of multiple countries. For strategic industries, many countries will directly intervene and soon formulate domestic reserve plans and supply guarantee systems.

Zhejiang Province is a big market Province in China's open economy. The specialized market was once a major institutional innovation in Zhejiang's reform and opening up. Due to this influence, the economic cycle chain of the specialized market was blocked, and there are problems at both ends of supply and demand. Foreign trade was changing from insufficient supply to declining demand. Supply shortages of products or raw materials, transportation delays, containers, and emergencies will be important challenges for industrial chain/supply chain disruption. It was urgent to make up for the weakness through supply chain innovation; comply with the new changes in consumption mode, investment demand, production organization mode, and market competition at home and abroad; pay attention to the overall construction of the global industrial chain supply chain; strengthen the transformation from the original elements to investment driven and to innovation driven; and seek a new path of transformation and innovation development.

The article "Bayesian Estimation of Supply Chain Innovation Path" was retracted in 2023. Reasons: unreliable results or conclusions; concerns about the data; concerns about the peer review; concerns about the citations.

The concept of supply chain innovation can be traced back to Joseph Alois Schumpeter and Drucker's innovation theory. Therefore, innovation can be divided into three categories: one was based on Schumpeter's theory of technological innovation, the second was based on Schumpeter's theory of organizational innovation, and the third was based on Drucker's management tool theory.

Based on Schumpeter's theory of technological innovation, supply chain innovation was the combination of information technology or supply chain technology and other production factors, which aimed to improve operational efficiency, increase revenue, create value, etc. At present, the concept proposed was most cited by scholars. Ernest et al. believed that supply chain innovation was a combination of information technology, new marketing, and logistics process, whose purpose was to improve service efficiency, improve operation efficiency, increase revenue, and maximize common profit [1].

Supply chain innovation was not only the recombination of production factors but also a dynamic process. Zhong believed that supply chain innovation was a change in supply chain network, supply chain technology, or supply chain process (or a combination of the three). This kind of change occurred in the company's functional departments, within the company, industry, or supply chain, in order to promote the new value creation of stakeholders [2] Obviously, Jan stentoft's definition was consistent with Schumpeter's “innovation is a revolutionary change,” and “innovation must be able to create new value.” Compared with the concept proposed by Dahlmann and Roehrich, Jan stentoft emphasizes the dynamic nature of supply chain innovation. Furthermore, Kusi-Sarpong et al. believed that supply chain innovation was to develop new technologies and procedures and implement new ideas of products and services through necessary supply chain activities. At the same time, supply chain innovation was a kind of dynamic ability of enterprises because it could make enterprises produce more value-added products and services as well as stronger competitiveness [3, 4].

The article "Bayesian Estimation of Supply Chain Innovation Path" was retracted in 2023. Reasons: unreliable results or conclusions; concerns about the data; concerns about the peer review; concerns about the citations.

Based on Schumpeter's organizational innovation theory, supply chain innovation was a process in which supply chain partners promote innovation through collaboration and information exchange rather than the self-innovation of an enterprise. When the focus enterprise, suppliers, retailers, and customers were committed to innovation, supply chain innovation performance could be improved. Therefore, supply chain innovation was a cross-organizational innovation. Juliet and Liu believed that logistics, which was an important part of the supply chain, required close and coordinated information exchange between supply chain partners. In this sense, the process of supply chain innovation was a cross-organizational and distributed innovation process [5]. Hau and others believed that supply chain innovation was a complex process that used new technologies to deal with environmental uncertainty and respond to customer needs and improved organizational processes in new ways [6]. Aamer believed that supply chain innovation was a relational, a cross-cultural, and cross-organizational phenomenon, and this success will eventually lead to continuous innovation [7]. It was not difficult to see that from the perspective of organizational innovation, it emphasized that supply chain innovation was the result of the joint efforts of many organizations in the supply chain. They deal with the environmental uncertainty through information exchange and close coordination and promote the innovation of the supply chain organizational form.

Based on Drucker's management tool theory, supply chain innovation was a kind of management tool, which can improve the operation process of the supply chain and promote the interaction and sharing between focus enterprises and suppliers, retailers, and customers so as to achieve efficient supply chain management. Lin and Lee put forward a highly consistent concept. Phan and others described supply chain innovation as a set of tools, which can improve enterprise processes through seamless integration with suppliers, manufacturers, distributors, and customers so as to achieve efficient supply chain management. [8].

In the dimension of supply chain innovation, there were more three-dimensional models of supply chain innovation. The most representative is the three-element interaction model constructed by Bodlaj and Mateja. They believed that supply chain innovation was formed by the interaction of three factors, namely, supply chain business process, supply chain network structure, and supply chain technology. These three elements were not static but triggered by the dynamic interaction between the enterprise and its business environment. They interact in the dynamic cycle of enterprise business model change and innovation [9]. The first mock exam was Carnovale et al. which was a case study. The model was composed of three interrelated parts: supply chain technology, supply chain business process, and supply chain network structure [10]. The model constructed by Jan stentoft showed that supply chain innovation was a dynamic process, and “process” was an important content of supply chain innovation as well as “technology.” Ganguly, Anirban divided supply chain innovation into three dimensions: supply chain innovation objectives, supply chain characteristics, and innovation characteristics. It constructed a theoretical foundation for the follow-up research [11].

The article "Bayesian Estimation of Supply Chain Innovation Path" was retracted in 2023. Reasons: unreliable results or conclusions; concerns about the data; concerns about the peer review; concerns about the citations.

Overviewing the existing literature, the classification of supply chain innovation was basically based on the concept of technology innovation theory. In particular, the supply chain technology innovation was regarded as an important category of supply chain innovation. According to Campello, Murillo's study (2017), it divided supply chain innovation into supply chain concept innovation and supply chain technology innovation [12]. Among them, conceptual innovation of the supply chain included structural innovation, operational innovation, and revolutionary innovation. Structural innovation led to the change in the supply chain structure, operational innovation aimed to improve logistics, and revolutionary innovation led to the profound change in the supply chain structure and operation. Supply chain technology innovation improved the efficiency of information and material exchange in the supply chain [13]. According to the concept of Stylianos and Karl, Tseng et al. divided supply chain innovation into three key innovation activities: logistics-oriented innovation activities, marketing-oriented innovation activities, and technology development-oriented innovation activities. Among them, logistics-oriented innovation activities were innovative services related to logistics. Such services were beneficial to target customers, which could be external or internal. For external target customers, innovation can better serve customers, and for internal target customers, innovation can improve operation efficiency. Marketing-oriented innovation activities were innovative services related to marketing, and its purpose was to meet the needs of customers. Technology development-oriented innovation activities include creating new knowledge and new technical skills and developing new services/products for customers [14].

The article "Bayesian Estimation of Supply Chain Innovation Path" was retracted in 2023. Reasons: unreliable results or conclusions; concerns about the data; concerns about the peer review; concerns about the citations.

To sum up, relevant scholars have discussed the basic concepts, dimensions, and types of supply chain innovation. However, as a low-cost and low-risk market, there are still many problems to be further clarified, such as how the supply chain quickly corresponds to the complex innovation network system, or where the supply chain innovation should start.

## 2. Supply Chain Innovation Path

Supply chain refers to a functional network chain structure that centers on the core enterprise, starting from supporting parts, making intermediate products and final products, and finally sending products to consumers by the sales network, connecting suppliers, manufacturers, distributors, and end users as a whole. It was a complex network chain structure composed of logistics, business flow, capital flow, and information flow, which was composed of multilevel enterprises across organizational boundaries, industries, and many nodes, and had different products, services, technologies, and business models (Figure 1). Different from the innovation decision-making within a single enterprise organization, cross-organizational boundaries were affected by the demands of different stakeholders, and the innovation decision-making was more complex. One of the important decisions was who will lead the innovation drive and where and when to start. Supply chain innovation decision and its implementation process were a complex system engineering. In order to improve and meet the market demand as the core, the benefit maximization of the whole supply chain is realized. It requires not only the supply chain to maintain the self-height service level but also the coordination of service between the supply chain. The whole process was full of the continuous innovation game of competition and cooperation. Cooperation and competition had their own characteristics. Cooperation could effectively coordinate interpersonal relationships and improve work efficiency. However, in the process of cooperation, there was also competition among group members, which played a significant role in improving personal work efficiency. In addition, when a group cooperates, it must compete with other members. Therefore, competition and cooperation are interdependent and indispensable. Competition and cooperation at the supply chain level mainly focus on the supply chain strategy level. The focus of supply chain strategy is the market value created by the process of products or services moving within the enterprise and the whole supply chain. The focus has shifted from inward capabilities to integrating their capabilities with production resources and innovation knowledge in supply chain members. Cooperation cannot be without competition within the supply chain. Cooperation without competition is a backwater. When competition was in cooperation, competition could better achieve the goal. Competition could not be without cooperation. Competition without supply chain cooperation was lonely, and lonely competition was powerless. There must be both competition and cooperation among supply chain entities. It had the sustainability and vitality in the supply chain.

The article "Bayesian Estimation of Supply Chain Innovation Path" was retracted in 2023. Reasons: unreliable results or conclusions; concerns about the data; concerns about the peer review; concerns about the citations.

Therefore, in view of the demand of supply chain innovation, we must establish a new analysis framework structure, which was guided by market demand and connects various current information flows so as to better tap the internal motivation of innovation in the supply chain. From the perspective of supply chain competition, first of all, it determines the products/services that the supply chain can meet the future market. Then, combined with the current situation of the supply chain, it analyzes the tasks and assets (capabilities) that transform the product/service demand into processes and various subprocesses, and obtains the relevant influencing factors of supply chain innovation. With the help of these factors, we can improve the accuracy of supply chain innovation-driven forecasting to ensure the success of innovation. In fact, the Bayesian model can effectively use all available data to diagnose consumer preferences and express the relevant information as a set of relationships among variables [15, 16]. Therefore, this study constructs a Bayesian model of supply chain innovation path dependence and establishes a market-oriented supply chain innovation decision-making framework. Bayesian model is also called the belief network model. Bayesian model can be regarded as a directed acyclic graph, which is composed of nodes representing variables and directed edges connecting these nodes. A node represents a random variable, and the directed edge between nodes represents the relationship between nodes (from the parent node to its child node). Conditional probability is used to express the relationship strength, but no parent node uses a priori probability to express the relationship between information [17]. Each node *C* has a probability distribution, which represents the uncertainty of related variables, where *f*(*c*) represents the previous node of node *C* (if *f*(*c*) in node *C*) = *ø*, represents a nonparent node). Therefore, under the assumption of independence, n-node Bayesian network (*C*1, *C*2,..., *CN*) can be expressed as a joint probability distribution:

(1) $$\begin{array}{c} P\left(c_{1},\ldots ,c_{n}\right)=\prod_{i=1}^{n}p\left(c_{i}|f\left(c_{i}\right)\right). \end{array}$$

The results of the model can reveal the individual innovation ability and intensity of supply chain innovation. As part of the innovation decision, finally, through sensitivity analysis, we can determine which variables significantly affect consumer preference. *IE* (information exchange) can measure the dependence between two random variables, which is suitable for sensitivity analysis of Bayesian networks. If we know the variable *V*1, we can reduce the uncertainty of variable *V*2. The *IE* between variables can be expressed as

(2) $$\begin{array}{c} IE\left(v_{1},v_{2}\right)=\sum P\left(v_{1},v_{2}\right)\text{log}\frac{P\left(v_{1},v_{2}\right)}{P\left(v_{1}\right)P\left(v_{2}\right)}, \end{array}$$

where *P* (*V*1, *V*2) is the joint probability distribution, *P* (*V*1) is the probability distribution function of *V*1, and *P* (*V*2) is the probability distribution function of *v*2. *IE* (*V*1, *V*2) represents the interaction between variables *V*1 and *V*2. The larger the value is, the closer the relationship between variables *V*1 and *V*2 is. Therefore, the importance of variables can be judged according to the size of *IE* (*V*1, *V*2). In practice, the larger the (*V*1, *V*2), the more relevant variables need to be concerned. In addition, the Bayesian network can reflect the changing market demand in time, and each node organization in the supply chain can drive the continuous innovation of products/services through continuous improvement of Bayesian network.

The article "Bayesian Estimation of Supply Chain Innovation Path" was retracted in 2023. Reasons: unreliable results or conclusions; concerns about the data; concerns about the peer review; concerns about the citations.

With the help of the above model, each node of the supply chain was allowed to merge its own capability set with other nodes. By linking resource capability set from different nodes, the actual demand was subdivided into product design, production, sales, after-sales, and other processes, thus objectively determining the transmission process of innovation capability set required by product/service. It was assumed that AE is the problem to be solved in product/service innovation, TR was the ability set that is really needed, SK was the ability set that can be obtained to solve specific problems, and mediation skills (MT) can improve the learning speed or connect TR and SK models to help decision makers obtain TR from SK. The basis of this method is to try to build an inference network graph (SK) from the starting node, from the beginning to the middle node (MT) to the end node (TR), and then use 0-1 integer programming to find the optimal solution. Because the data of internal capability (MT), existing capability set (SK), required capability set (TR), habit domain of related skills, and learning cost can be obtained by using data mining technology, these data can be input into the reasoning diagram; thus, a specific mathematical model of supply chain innovation behavior evolution mechanism based on Bayesian model can be constructed. The corresponding optimal solution can be obtained. The optimal solution shows how the whole innovation capability set of the corresponding supply chain is transformed into the whole supply chain process according to the market demand and is refined into the tasks and assets of the supply chain members.

The article "Bayesian Estimation of Supply Chain Innovation Path" was retracted in 2023. Reasons: unreliable results or conclusions; concerns about the data; concerns about the peer review; concerns about the citations.

## 3. Empirical Study

This project selects 5 kinds of products/services *P* (*p* = (*P*1,... *P*5) with different market demands based on the Bayesian model based on the supply chain with a professional market in Zhejiang as the core collected in the early stage and identifies the capability set required by each product/service (Table 1). *AE*(*AE* = (*a*1,…, *a*14)) represents different capability sets. Assume the following:

1. Different products/services require different sets of capabilities. For example, product/service *P*1 needs capability set {ai}, while product/service *P*2 needs capability set {aj}.
2. As the core of the supply chain, the professional market has two channels to choose from which are as follows: SC1 and SC2. Channel SC1 has *A*3, *A*4, and *A*5 capability sets; channel SC2 has capability sets *A*1, *A*2, and *A*6. It is easy to know that neither channel SCI nor channel SC2 can provide the required feature set for all products/services alone. In order to provide corresponding products/services, each channel needs to learn the existing capability set to obtain a new capability set. For example, suppose that the selling price of capability set *A*3 is 0.4 units and that of capability set *A*6 is 0.6 units.
3. The cost for channel SC1 to obtain the innovation capability set is shown in Table 2, and the cost for channel SC2 to obtain the innovation

capability set is shown in Table 3 (for consistency, the maximum cost is one unit for ex weighting). It is found that channel SC1 and channel SC2 should focus on different products/services. Considering the acquisition cost of the capability set, channel SC1 should focus on product/service *P*1, *P*2, and *P*3; channel SC2 should focus on product/service *P*4 and *P*5. Assuming that channel SCI and channel SC2 can only provide one product/service, respectively, there will be six product/service combinations as shown in Table 4 (for the convenience of calculation, the data are integer and dimensionless).

The capacity set network diagrams of channels SC1 and SC2 are constructed, respectively, as shown in Figures 2 and 3. Each node represents a capability set, and the edge represents the relationship between capability sets.

The article "Bayesian Estimation of Supply Chain Innovation Path" was retracted in 2023. Reasons: unreliable results or conclusions; concerns about the data; concerns about the peer review; concerns about the citations.

For example, *A*5 to *A*6 indicate that the capability set *A*6 can be obtained through the learning capability set *A*5. If there is no edge between nodes *A*13 and *A*7, the capability set *A*13 cannot be obtained through the learning capability set *A*7 and vice versa. The value of the edge shows the innovation cost of acquiring a new capability set. In addition, there are composite nodes, such as *A*4 ^ *A*5 and *A*1 ^ *A*2, which are composite function sets. It should be noted that when using composite nodes, each child node must exist. For example, SC2 channel can only use a composite capability set if it has both *A*1 and *A*2 capability sets a1^a2. In order to provide corresponding products/services, we need to acquire other capabilities. For example, online channels can purchase from offline channels or learn from existing capability sets to acquire new capability sets. In fact, for ability set a3, channel SC2 can be obtained by learning ability set a6, a1^a2, a1, or purchased from channel SC2. Of course, the cost of acquisition was 0.6, 0.4, 0.72, and 1. In short, the ultimate goal of building the above capacity set network diagram is to find out the best product/service combination by using optimization method so as to maximize the overall profit of the supply chain. Taking the minimum cost flow of the whole supply chain as the objective function, the optimal products/services of SC1 and SC2 were obtained. For SC1, the best product/service is *P*1. To provide *P*1 products/services, channel SC1 needs to pay 5 units to obtain the capability set {*a*6, *a*7}. The channel SC1 was expected to get the expected profit of 11 units under the optimal condition. For SC2, the best product/service was *P*4. To provide *P*4 products/services, channel SC2 needs to pay 3.6 unit cost to obtain the capability set {*a*3, *a*10}. Get the expected return of 9 units. It was expected that channel SC2 will get 5.4 units of expected profit under the optimal situation. For the whole supply chain, what is the optimal product/service combination {*p*1, *p*4}. It was expected that the supply chain will obtain the expected profit of 16.4 units. To sum up, we use the Bayesian model to subdivide the market demand for products/services, to make clear what kind of best products/services the supply chain can provide, and how to obtain market revenue through innovation, which provides a more reliable decision-making basis for enterprises in the supply chain to make supply chain innovation decisions.

The article "Bayesian Estimation of Supply Chain Innovation Path" was retracted in 2023. Reasons: unreliable results or conclusions; concerns about the data; concerns about the peer review; concerns about the citations.

## 4. Conclusion

Supply chain innovation was different from pure technological innovation, management innovation, and innovation of other organizations. Supply chain innovation was more innovation across organizational boundaries. The supply chain innovation path beyond the organizational boundary was a difficult problem that must be solved at the macro- and microlevel. However, it was very clear that there were many ways for supply chain innovation, which can only be completed on the basis of certain materials. This study abstracted the material base to the capability set of each node company in the supply chain, calculated the difference between incremental and stock capabilities, judged the urgency and difficulty of supply chain innovation by the difference, and put forward the supply chain innovation path theory. This paper made an empirical study on the supply chain with specialized market which provided a better solution for supply chain innovation decision-making. The research results of the supply chain innovation path were obtained based on the assumption that the overall interests of the supply chain are consistent. Because of well known, the asymmetry of information and the market was not clear. So, if the demands of various stakeholders of the supply chain were not consistent, the decision-making of supply chain innovation will become more complex and difficult. Therefore, when the market has not been completely cleaned up, how to solve the supply chain innovation decision-making will be an in-depth research topic in the future.

## Figures and Tables

**Figure 1:** Basic structure of supply chain.

**Figure 2:** SC1 capability set network diagram.

**Figure 3:** SC2 capability set network diagram.

**Table 1:** Market demand supply chain capability response.

	*a*1	*a*2	*a*3	*a*4	*a*5	*a*6	*a*7	*a*8	*a*9	*a*10	*a*11	*a*12	*a*13	*a*14
*P*1	—	—	—	—	—	√	√	—	—	—	—	—	—	—
*P*2	—	—	—	—	—	√	√	—	√	—	—	—	—	—
*P*3	—	—	—	√	—	—	—	√	—	—	—	—	√	√
*P*4	—	√	√	—	—	—	—	—	—	√	—	—	—	—
*P*5	—	—	—	—	—	√	—	—	—	—	√	√	—	—

**Table 2:** Cost of SC1 acquiring innovation capability set in supply chain.

	_*a*6_	_*a*7_	_*a*8_	_*a*9_	_*a*13_	_*a*14_
_*a*3_	_1_	_0.6_	—	_0.4_	—	—
_*a*4_	—	—	_1_	_0.6_	—	—
_*a*5_	_1_	—	—	—	_0.4_	—
_*a*4 ^*a*5_	_0.4_	—	_0.4_	—	—	_0.6_
_*a*6_	—	_0.4_	—	—	—	_1_
_*a*7_	—	—	—	_0.6_	—	—
_*a*8_	—	—	—	—	—	_1_
_*a*9_	—	_0.4_	—	—	—	—
_*a*13_	—	—	—	—	—	—
_*a*14_	_0.4_	—	_0.72_	—	—	—

*Note*. “—” indicates that there is no interaction.

**Table 3:** Cost of SC2 acquiring innovation capability set in supply chain.

	_*a*3_	_*a*10_	_*a*11_	_*a*12_
_*a*1_	_0.72_	—	_1_	—
_*a*2_	—	—	_0.72_	—
_*a*1^*a*2_	_0.4_	—	_0.6_	—
_*a*3_	—	_0.4_	—	—
_*a*6_	_0.6_	_0.4_	—	_0.4_
_*a*10_	_0.4_	—	—	—
_*a*11_	—	—	—	_0.4_
_*a*12_	—	_0.6_	—	—

*Note*. “—” indicates that there is no interaction.

The article "Bayesian Estimation of Supply Chain Innovation Path" was retracted in 2023. Reasons: unreliable results or conclusions; concerns about the data; concerns about the peer review; concerns about the citations.

**Table 4:** Expected return of product/service portfolio.

_Product/service mix_	_SC1_	_SC2_
_*p*1,*p*4_	_16_	_9_
_*p*1,*p*5_	_14_	_10_
_*p*2,*p*4_	_11_	_8_
_*p*2,*p*5_	_12_	_7_
_*p*3,*p*4_	_10_	_6_
_*p*3,*p*5_	_8_	_7_

## Data Availability

Data sharing is not applicable to this article as no data sets were generated or analysed during the current study.
